The article "Electrostrictive and Structural Properties of Poly(Vinylidene Fluoride-Hexafluoropropylene) Composite Nanofibers Filled with Polyaniline (Emeraldine Base)" was published in 2021. Journal: Polymers (Basel).

# Electrostrictive and Structural Properties of Poly(Vinylidene Fluoride-Hexafluoropropylene) Composite Nanofibers Filled with Polyaniline (Emeraldine Base)

**DOI:** 10.3390/polym13193250

**Published:** 2021-09-24

**Authors:** Nikruesong Tohluebaji, Chatchai Putson, Nantakan Muensit, Jureeporn Yuennan

**Affiliations:** 1 Faculty of Science and Technology, Princess of Naradhiwas University, Narathiwat 96000, Thailand; nikruesong.t@pnu.ac.th; 2 Center of Excellence in Nanotechnology for Energy (CENE), Division of Physical Science (Physics), Faculty of Science, Prince of Songkla University, Songkhla 90112, Thailand; chatchai.p@psu.ac.th (C.P.); nantakan.m@psu.ac.th (N.M.); 3 Surface Technology Research Unit (STRU), Faculty of Science and Technology, Nakhon Si Thammarat Rajabhat University, Nakhon Si Thammarat 80280, Thailand

**Keywords:** electrostrictive, poly(vinylidene fluoride-hexafluoropropylene), polyaniline, nanofibers

## Abstract

Previous studies have reported that poly(vinylidene fluoride-hexafluoropropylene) (P(VDF-HFP)) copolymers can exhibit large electrostrictive strains depending on the filler. This work examines the electrostrictive and structural properties of P(VDF-HFP) nanofibers modified with conductive polymer polyaniline (PANI). The P(VDF-HFP)/PANI composite nanofibers were prepared by an electrospinning method with different PANI concentrations (0, 0.5, 1, 1.5, 3 and 5 wt.%). The average diameter, water contact angle and element were analyzed by SEM, WCA and EDX, respectively. The crystalline, phase structure and mechanical properties were investigated by XRD, FTIR and DMA, respectively. The dielectric properties and electrostrictive behavior were also studied. The results demonstrated that the composite nanofibers exhibited uniform fibers without any bead formation, and the WCA decreased with increasing amount of PANI. However, a high dielectric constant and electromechanical response were obtained. The electrostrictive coefficient, crystalline, phase structure, dielectric properties and interfacial charge distributions increased in relation to the PANI content. Moreover, this study indicates that P(VDF-HFP)/PANI composite nanofibers may represent a promising route for obtaining electrostrictive composite nanofibers for actuation applications, microelectromechanical systems and sensors based on electrostrictive phenomena.

## 1. Introduction

Electroactive polymers (EAPs) are materials that respond to electrical stimulation by exhibiting significantly large strains. EAPs have gained tremendous attention from researchers worldwide because of their attractive merits of large bending deformation, quick response, thinness, flexibility, relatively low cost and light weight [1,2]. Among the known EAPs, poly(vinylidene fluoride) (PVDF) and its copolymers, such as polyvinylidenefuoride hexafuoropropylene (P(VDF-HFP)), have been widely studied due to their relatively large and fast electromechanical response, high breakdown strength, high mechanical and chemical stability, flexibility, low acoustic impedance, low cost and also processing advantages. Therefore, they have been extensively used for a wide range of applications, such as sensors, actuators, energy harvesting and biomedicine [3,4]. Previously, it has been reported that the piezoelectric coefficient (d_31_), electromechanical coupling factor (k_31_) and dielectric constant in P(VDF-HFP) are higher than those of a PVDF homopolymer [5].

The article "Electrostrictive and Structural Properties of Poly(Vinylidene Fluoride-Hexafluoropropylene) Composite Nanofibers Filled with Polyaniline (Emeraldine Base)" was published in 2021. Journal: Polymers (Basel).

P(VDF-HFP) is a semi-crystalline polymer that consists of a repeating unit of the CH_2_CF_2_ monomer and commonly exists in at least four crystal forms, namely α-, β-, γ- and δ-phases. Among these polymorphs, the β-phase (*all-trans* (TTTT) conformation) is the most polar form and is responsible for the piezo-, pyro- and ferroelectric properties due to its large spontaneous polarization [6]. Over the years, while numerous strategies have been developed to promote the electroactive polar β-phase in P(VDF-HFP), an electrospinning process has attracted attention as it provides high orientation of the polymer chains under an applied high electric field. It is simple, versatile, practical, inexpensive and offers promising characteristics for the fabrication of uniform and ultrafine fibers. Electrospun nanofibers with unique characteristics, such as high aspect ratio, large surface area, excellent porosity and light weight, have been achieved [7,8]. Najjar et al. [9] successfully fabricated P(VDF-HFP) nanofibers on flexible substrates in a novel biocompatible device, which demonstrated high mechanical-to-electrical conversion performance, with stretched P(VDF-HFP) nanofibers outperforming regular electrospun samples by more than 10 times. The stretched nanofibers had a higher β-phase content. Moreover, composite P(VDF-HFP) nanofibers have attracted widespread attention from the scientific community. Pi et al. [10] fabricated multi-structured SiO_2_@P(VDF-HFP) nanofibrous membranes with a smaller fiber diameter and larger porosity. The SiO_2_@P(VDF-HFP) nanofibrous membranes also formed a superhydrophilic surface with a contact angle near to 0◦. Ponnamma et al. [11] designed a highly flexible piezoelectric nanogenerator (PENG) using PVDF and P(VDF-HFP) composite nanofibers filled with two nanostructured semiconducting metal oxides: nanotubes of TiO_2_ and nanoflowers of ZnO. The research showed that the composite nanofiber mats, with excellent mechanical strength, ligh weight and flexibility, are capable of producing a good output voltage (a maximum of 14 V) during different mechanical vibrations at various frequencies and in response to human motion. Our group previously demonstrated that P(VDF-HFP)/ZnO composite nanofibers exhibit a strain response and energy-harvesting capabilities. The electrostriction coefficient tended to increase with higher ZnO content and an increasing dielectric constant. The generated current increased with the ZnO content when the external electric field was applied at a vibration of 20 Hz [12]. Currently, polyaniline (PANI), considered one of the most popular conductive polymers, has been reported as a conducting component in P(VDF-HFP) composite to enhance the electrical properties due to its unique electrical and electrochemical properties, ease of synthesis and high environmental stability [13]. However, the P(VDF-HFP)/PANI composite prepared by the electrospinning process has rarely been reported in the literature.

The article "Electrostrictive and Structural Properties of Poly(Vinylidene Fluoride-Hexafluoropropylene) Composite Nanofibers Filled with Polyaniline (Emeraldine Base)" was published in 2021. Journal: Polymers (Basel).

The aim of the present work is to improve the dielectric and electrostrictive properties of P(VDF-HFP) nanofibers with the addition of PANI. P(VDF-HFP)/PANI composite nanofibers with various PANI concentrations are fabricated by the electrospinning method. The influence of the PANI filler on the surface morphology, crystallinity, phase structure, mechanical properties and electrical and electrostrictive properties of as-received nanofibers samples are investigated.

## 2. Materials and Methods

### 2.1. Materials and Composite Nanofiber Preparation

Poly(vinylidene fluoridene-hexafluoropropylene) (P(VDF-HFP); Solef 11010/1001, Solvay Solexis, Inc., Albright, WV, USA) powder and N, N-dimethylformamide (DMF; D158550, Sigma-Aldrich, St. Louis, MO, USA) were used as a polymer matrix and solvent, respectively. The P(VDF-HFP) powder was dried at 60 °C for 6 h prior to being used. Polyaniline (PANI; emeraldine base; 576379, Sigma-Aldrich) was used as a filler doped into the neat polymer solution.

The P(VDF-HFP)/PANI composite nanofibers were fabricated by a simple electrospinning method. Firstly, 5 g dried P(VDF-HFP) powder was dissolved in 20 mL DMF solvent and kept continuously under a magnetic stirrer at 40 °C, stirring until a transparent solution was achieved. Thereafter, the PANI filler was mixed into the P(VDF-HFP) solution by adjusting the weight percent to 0.0, 0.5, 1.0, 1.5, 3.0 and 5.0 wt.%. The whole mixture was magnetically stirred for 2 h to achieve a homogeneous mixture. Next, each viscous solution was loaded into a 20 mL plastic syringe connected to a stainless-steel needle, as shown in Figure 1a. Figure 1b shows the electrospinning setup to prepare pure P(VDF-HFP) and P(VDF-HFP)/PANI composite nanofibers. The solution was electrospun in the horizontal direction at a flow rate of 0.5 mL/h, controlled by a syringe pump (Nz1000 NEWERA Pump Systems Inc., New York, NY, USA). The distance from the tip (positive pole) to the collector (negative pole) was fixed at 20 cm and the applied voltage was 17 kV using a high-voltage supply (PHYWE Item No. 13671-93, Göttingen, Germany). Finally, the pure P(VDF-HFP) and P(VDF-HFP)/PANI composite nanofibers were obtained on an aluminum foil substrate pasted onto the collector.

The article "Electrostrictive and Structural Properties of Poly(Vinylidene Fluoride-Hexafluoropropylene) Composite Nanofibers Filled with Polyaniline (Emeraldine Base)" was published in 2021. Journal: Polymers (Basel).

### 2.2. Material Characterization

#### 2.2.1. Surface Morphology, Water Contact Angle and Elemental Analyses

The surface morphology of all the nanofibers was investigated using a scanning electron microscope (SEM; FEI Quanta 400, The Netherlands). Each sample was processed at a magnification of 1000× and 10,000×. To explore the wettability of the nanofibers’ surfaces, the fiber diameters of all samples were determined, which also resulted in a change in their water contact angle. The average diameter was determined from the SEM image using the ImageJ processing software (ImageJ; National Institutes of Health, 1.46, Bethesda, MD, USA). The water contact angle of the surface was also characterized using the Dataphysics Contact Angle System (OCA-15EC, Filderstadt, Germany) in static sessile drop mode. Energy-dispersive X-ray (EDX; X-stream-2, Oxford, UK) was used for the analysis of the elemental components of the samples. The elemental mapping signal of each sample was used to determine the chemical components on the surface, such as fluorine (F) and carbon (C).

#### 2.2.2. Crystalline and Phase Structure Investigations

The crystallinity of pure and composite nanofibers was investigated using an X-ray diffractometer (XRD; X’Pert MPD, Philips, Amsterdam, The Netherlands) in the 2θ range of 5° to 90° at a scanning rate of 0.05°/1 s. The percentage crystalline degree (*X_c_*) of the sample could be calculated according to Equation (1) [14]:

(1) $$X_{c}=\frac{\Sigma A_{Cr}}{\Sigma A_{Cr}+\Sigma A_{amr}}\times 100\%,$$

where $\Sigma A_{Cr}$ and $\Sigma A_{amr}$ are the total value of the integral area of crystalline diffraction peaks and amorphous, respectively. Moreover, the phase structure of all samples was considered using a Fourier transform infrared spectrometer (FTIR; Vertex70, Bruker, Germany) in the range of 400–2000 cm^−1^. The fraction of β-phase [F(β)] was given by Equation (2) [15]:

(2) $$F(\beta )=\frac{A_{\beta }}{\left(\frac{k_{\beta }}{k_{\alpha }}\right)A_{\alpha }+A_{\beta }}=\frac{A_{\beta }}{1.26A_{\alpha }+A_{\beta }},$$

where *A_β_* and *A_α_* are the absorption peaks of the crystalline phase at 840 and 763 cm^−1^, respectively. The number 1.26 is the ratio of the absorption coefficients at 840 and 763cm^−1^. The absolute β fraction (%β) was calculated by Equation (3) [16].

(3) $$\%\beta =F(\beta )\times X_{c}$$

The article "Electrostrictive and Structural Properties of Poly(Vinylidene Fluoride-Hexafluoropropylene) Composite Nanofibers Filled with Polyaniline (Emeraldine Base)" was published in 2021. Journal: Polymers (Basel).

#### 2.2.3. Dynamic Mechanical and Young’s Modulus Analyses

Dynamic mechanical analysis (DMA; Perkin Elmer, Groningen, The Netherlands) can be used to identify the storage modulus (*E*′), loss modulus (*E*) and tan delta (*tanδ*). The DMA testing was performed from −100 to 140 °C with a heating rate of 5 °C/min at a constant frequency of 1.0 Hz. Furthermore, Young’s modulus (*Y*) was investigated to determine the longitudinal strain (*S*_33_) based on the sizeable mechanical deformation in the electrostriction application. The modulus of all samples was measured by a strain gauge setup with a force gauge (BFG50N, Mecmesin, West Sussex, UK). Rectangular samples were cut from the original sheets with a size of 5 × 30 mm^2^. The modulus of the samples was calculated from the slope of the stress (*σ*)–strain (*ε*) curve on the elastic region (*ε* < 5%). 

#### 2.2.4. Dielectric Properties and Electrostriction Behavior

The dielectric constant (*ε_r_*) and loss tangent (*tanδ*) of P(VDF-HFP) nanofibers with different PANI concentrations were evaluated as a function of applied frequency in the range of 10^2^–10^5^ Hz using an LCR meter (IM 3533, HIOKI, Nagano, Japan) at room temperature. For electrostrictive measurement, each P(VDF-HFP) nanofiber film was examined by measuring the electric field (*E*)-induced strain (*S*) with a photonic displacement sensor (MTI-2100 Fotonic sensor, Albany, NY, USA), as demonstrated in Figure 2. All samples were sandwiched between two brass electrodes, and the weight of the top brass disc was 5 g, which was advisable for small stress, to avoid clamping of the sample. The electric field-induced strain was applied along the thickness direction. The thickness deformation of all samples was determined using a photonic sensor and a lock-in amplifier (610E, Trek, Waterloo, WI, USA).

## 3. Results and Discussion

### 3.1. Surface Morphology

Figure 3 presents images of the specimens of pure P(VDF-HFP) and P(VDF-HFP)/PANI composite nanofibers at 0.0, 0.5, 1.0, 1.5, 3.0 and 5.0 wt.%. As the concentration of PANI increases, the color of the composite nanofibers changes from white to navy blue, which is the color of the PANI powder, indicating the presence of the additives in the composite. SEM images of pure P(VDF-HFP) and P(VDF-HFP)/PANI composite nanofibers are also shown in Figure 4. As can be observed in the SEM image of the pure P(VDF-HFP) nanofiber mat with 1000× magnification, a number of bead-on-string fibers are randomly produced. For composite fibers, when PANI concentrations are doped from 0.5 to 3.0 wt.%, the bead-on-string structures evidently disappear, which can be attributed to the higher conductivity in the composite solution during the electrospinning process, as previously considered by Uyar T., et al. [17]. Remarkably, the structure of 5.0 wt.% P(VDF-HFP)/PANI composite is composed of bead-free, continuous and aligned fibers. This observation can be explained by the fact that the addition of the conductive PANI polymer results in stronger electrostatic repulsion, which reduces the surface tension forces, favoring the stretching of fibers to form the aligned fibers [18]. 

The article "Electrostrictive and Structural Properties of Poly(Vinylidene Fluoride-Hexafluoropropylene) Composite Nanofibers Filled with Polyaniline (Emeraldine Base)" was published in 2021. Journal: Polymers (Basel).

The SEM images were also used to analyze the average fiber diameter using the ImageJ program. As demonstrated in Table 1, the diameters of all fiber samples are observed in the nanoscale range. The incorporation of PANI content into P(VDF-HFP)/PANI composite nanofibers results in an increase in the diameter of the nanofiber. The diameter of the pristine P(VDF-HFP) nanofiber is 120.3 ± 20.6 nm, which then increases from 265.5 ± 53.1 to and 326.5 ± 99.5 nm after adding PANI from 0.5 to 5.0 wt.%, respectively. The enlarged diameter of the composite nanofibers may be caused by the PANI absorbed by the P(VDF-HFP) nanofibers mats, which is similar to the result previously reported by Dognani G., et al. [19]. The average diameter of the composite nanofibers increases with increasing PANI concentration due to the higher viscosity of the solutions after adding PANI. The water contact angle in pristine P(VDF-HFP) nanofibers is approximately 139.2 ± 3.2°, which then slightly decreases with the increasing amount of PANI in the composite, as shown in Table 1. This result is due to the inherent hydrophilic property of PANI, which contains abundant amine groups and has a water contact angle of 51.5° [20]. However, PANI filling is not sufficient to change the water contact angle of composite nanofibers, which still presented a hydrophobic surface (90° ≤ θ ≤ 150°). These composite nanofibers are suitable for some applications that are poor wettability. Moreover, the EDX spectra were recorded in order to study the chemical composition of the nanofibers. In Table 1, we show the weight percentage and atomic percentage of F and C elements existing in the nanofiber samples. The result confirms the presence of C and F elements originating from the pure P(VDF-HFP) copolymer. After loading PANI into the P(VDF-HFP) composite, the F element is reduced and the C element is increased, corresponding to the chemical formula of the PANI [([C_6_H_4_NH]_2_[C_6_H_4_N]_2_)_n_] homopolymer added to the composite. 

The article "Electrostrictive and Structural Properties of Poly(Vinylidene Fluoride-Hexafluoropropylene) Composite Nanofibers Filled with Polyaniline (Emeraldine Base)" was published in 2021. Journal: Polymers (Basel).

### 3.2. Crystalline and Phase Structure Analysis

Figure 5 shows the XRD patterns of pure P(VDF-HFP) and P(VDF-HFP)/PANI composite nanofibers with different PANI contents. The characteristic reflection peaks of crystalline at 2θ = 18.3° (020) and 26.6° (021) corresponding to α-phase formation and the peaks at 2θ = 20.3° (020)/(100) and 35.5° (110)/(200) assigned to the β-phase are observed [21]. The peaks of the α-phase at 18.8° and 26.6° are obviously presented in pure P(VDF-HFP) nanofibers. After the addition of PANI in P(VDF-HFP), the peaks of the α-phase are completely diminished and two peaks of the β-phase at 20.3° and 35.5° appear, indicating the presence of the β-phase in the composite nanofibers. The high voltage applied during the electrospinning process contributed to aligning the electric dipoles in the P(VDF-HFP) solution, leading to the formation of the polar β-phase in the composite nanofibers [22]. As seen in Table 2, the degree of crystallinity (*X_c_*) of pure P(VDF-HFP) nanofibers is 48.40%, and it increases upon the addition of PANI filler. The composite fibers are molecularly oriented during the electrospinning. 

The electroactive β-phase in the nanofiber samples was further examined via FTIR spectra. Figure 6 presents the FTIR spectra of pure and P(VDF-HFP)/PANI composite nanofibers with different PANI concentrations in the region of 400 to 2000 cm^−1^. The vibrational bands at 534, 617, 765 and 976 cm^−1^ are determined to the characteristic peaks of the α-phase observed in the pure P(VDF-HFP) nanofiber web [23], indicating that it contains α-phase formation. With the accretion of PANI filler, the characteristic peaks of the α-phase are entirely diminished and the peaks of the β-phase as marked bands at 838, 1234 and 1276 cm^−1^ are increased. It can be inferred that with PANI loaded in P(VDF-HFP), not only is the α-phase reduced but also the β-phase is also induced in the composite nanofibers. In Table 2, the relative fraction of β-phase content (*F(β)*) with various concentrations of PANI filler is shown. It is found that the *F(β)* values increase from 73.53% to 85.79% when the minimum amount of PANI (0.5 wt.%) is added to P(VDF-HFP). The *F(β)* values slightly increase with the increasing amount of PANI filler. Furthermore, the absolute β fraction (%*β*), evaluated by Equation (3) using the XRD and FTIR results, gives information about the overall β-phase within the as-prepared nanofibers. It is evident that the %*β* values increase rapidly upon adding only 0.5 wt.% of PANI and then increase gradually with the PANI content. These observations denote the effect of varying PANI filler loaded into P(VDF-HFP) nanofibers prepared by electrospinning techniques, which can affect the orientation of the dipoles to promote β-phase formation [24]. 

The article "Electrostrictive and Structural Properties of Poly(Vinylidene Fluoride-Hexafluoropropylene) Composite Nanofibers Filled with Polyaniline (Emeraldine Base)" was published in 2021. Journal: Polymers (Basel).

### 3.3. Mechanical Properties

Figure 6 presents the (a) storage modulus ($E^{\prime }$), (b) loss modulus and (c) tan delta (tanδ) of pure P(VDF-HFP) and P(VDF-HFP)/PANI composite nanofibers using the DMA measurement. Moreover, the thermomechanical properties and glass transition temperature ($T_{g}$) can be observed. It is found that the storage modulus of all samples decreases with increasing temperature. The storage modulus of P(VDF-HFP)/PANI composite nanofibers is greater than that of pure P(VDF-HFP) nanofibers, which confirms the reinforcement effect at the molecule interfaces [25]. A slow reduction in *E*′ is observed from −40 °C to 0 °C, which is ascribed to the glass transition of P(VDF-HFP) [26]. This effect demonstrates that semiconductor nanofillers influence the glass transition temperature of the P(VDF-HFP) nanofibers. Figure 6c offers *tanδ* as a function of temperature for pure and composite nanofibers at varying concentrations of PANI filler. The first peak damping of the relaxation process provided the α-relaxation, which was related to the motion in a crystalline fraction, while the second peak relaxation process depicted the melting temperature [22]. Normally, the glass transition temperature of a polymeric material is determined from the peak of the *tanδ* curve [27]. The β-relaxation is associated with a dynamic glass transition in amorphous and other semicrystalline polymers. The damping combined with the β process appears to be comparatively high for the nanofiber with broad β-transition from −80 °C up to −20 °C and a maximum temperature at −50 °C. The glass transition temperatures are approximately −53, −54, −52, −52, −53 and −52 °C for 0, 0.5, 1.0, 1.5, 3.0 and 5.0 wt.% of PANI doping, respectively. Figure 6e displays the Young’s modulus of pure P(VDF-HFP) and P(VDF-HFP)/PANI composite nanofibers with various concentrations of PANI, which were evaluated from the slope of the stress–strain curves in the elastic region (Figure 6d). The elastic modulus increased after PANI loading due to the rule of mixing properties. The addition of a conductive filler is normally associated with an increase in the interfacial surface area in the mixed composite solution between the filler particles and the host matrix [28]. The Young’s modulus of the composite nanofibers tends to be stable for higher PANI concentrations (with low Young’s modulus for lower PANI concentration).

### 3.4. Dielectric Properties and Electrostrictive Properties

Figure 7a shows the dielectric constant ($\varepsilon_{r})$ as a function of frequency with various amounts of PANI in P(VDF-HFP) nanofibers. At a low frequency (10^2^ Hz), a high dielectric constant is observed and it decreases with increasing frequency. The dielectric constant is associated with free dipole vibration in an alternating field at low frequency. The dielectric constant increases with the PANI concentration, as listed in Table 3. The $\varepsilon_{r}$ value at 10^2^ Hz increases from 1.48 to 2.58 for the 5 wt.% P(VDF-HFP)/PANI composite nanofibers, which is around 1.74 times that of the pure P(VDF-HFP) nanofibers. Clearly, the PANI reduces air gaps and induces surface charges, causing strong Maxwell–Wagner interfacial polarization. Furthermore, the dielectric loss tangent increases with the PANI concentration from 0.00071 to 0.02403 at 10^2^ Hz. It is recommended for use in ferroelectric and dielectric applications.

The article "Electrostrictive and Structural Properties of Poly(Vinylidene Fluoride-Hexafluoropropylene) Composite Nanofibers Filled with Polyaniline (Emeraldine Base)" was published in 2021. Journal: Polymers (Basel).

Figure 7b presents the longitudinal strain ($S_{33}$) as a function of an external electric field ($E_{3}$) for pure and composite nanofibers at a frequency of 1 Hz. The electric field-induced strain is quadratically related to the applied electric field, which is demonstrated by $S_{3}=M_{33}E_{3}^{2}$ ($M_{33}$ is the apparent electrostrictive coefficient) and Maxwell stress [29]. The Maxwell stress effect involves electrostatic attractions and interactions with the charges on electrodes, expressed by $S_{3}=\varepsilon_{0}\varepsilon_{r}E_{3}^{2}/Y$. Here, $\varepsilon_{0}$ is the permittivity of free space, $\varepsilon_{r}$ is the permittivity, and *Y* is the Young’s modulus. According to a prior publication, the strain from Maxwell stress is minimal compared to the measured strain, and therefore the Maxwell stress effect can be neglected [30]. Hence, it can be assumed that the measured strain is due to only the electrostrictive effect. The electric field-induced strain increases when increasing the content of PANI, due to the increased interface charge in the structure. However, when the external electrical field is expanded above approximately 8 MV/m, the electrostrictive strain becomes saturated due to the saturation of the electric field-induced polarization [30]. Figure 7c exhibits the relationship between the strain ($S_{33}$) and the square of the applied electric field ($E_{3}^{2}$) due to the slope being equal to the electrostrictive coefficient. It is clearly demonstrated that the electrostriction of composite nanofibers is significantly heightened after filling with PANI. Table 3 lists the dielectric constant ($\varepsilon_{r}$), loss tangent and conductivity (*σ*) at 10^2^ Hz. The Young’s modulus (*Y*) and electrostrictive coefficients ($M_{33}$) for all conditions are also reported. The results show that $\varepsilon_{r}$, loss tangent, *σ*, *Y* and $M_{33}$ increase remarkably with PANI filler loading. It can be inferred that the improved electrostriction relates to the dielectric constant and Young’s modulus of the composite [29,31]. The increased permittivity with PANI content suggests an increase in the interfacial charges. Moreover, this study indicates that P(VDF-HFP)/PANI composite nanofibers may represent a promising route for obtaining electrostrictive composite nanofibers for actuation applications.

The article "Electrostrictive and Structural Properties of Poly(Vinylidene Fluoride-Hexafluoropropylene) Composite Nanofibers Filled with Polyaniline (Emeraldine Base)" was published in 2021. Journal: Polymers (Basel).

## 4. Conclusions

PANI incorporation into P(VDF-HFP) composite nanofibers can be performed successfully by electrospinning techniques. The P(VDF-HFP)/PANI composite nanofibers exhibit uniform fibers without any bead formation, with a high dielectric constant and electromechanical response. The water contact angle of the nanofibers is found to be in the range of 126 ± 2.8° to 139.2 ± 3.2°, indicating a hydrophobic surface. The synergistic effect of electrospinning and the addition of PANI to the P(VDF-HFP) composite nanofibers can enhance the crystallinity, β-phase content and absolute β fraction by approximately 55.49%, 89.22% and 49.51% for a 5.0% PANI concentration, respectively. The elastic modulus and dielectric constant also increase after PANI filling. Furthermore, the P(VDF-HFP)/PANI 5 wt.% composite nanofibers display the largest electrostrictive coefficient *M*_33_ of approximately 2.53 × 10^−14^ m^2^/V^2^.

The results indicate that PANI addition in P(VDF-HFP) nanofibers can improve the electrostriction behavior attributed to the crystalline, phase structure, dielectric properties and interfacial charge distributions. The electrostrictive coefficient increases related to the PANI contents. Moreover, the electrostrictive strain response improves under low electric fields. This study indicates that P(VDF-HFP)/PANI composite nanofibers may represent a promising route for obtaining electrostrictive composite nanofibers for actuation applications that are poor wettability.

## Figures and Tables

**Figure 1:** Schematic drawing of (**a**) preparation of homogeneous solution and (**b**) electrospinning setup.

**Figure 2:** The electrostrictive measurement setup.

**Figure 3:** Photograph images of pure P(VDF-HFP) and P(VDF-HFP)/PANI composite nanofibers (0.0, 0.5, 1.0, 1.5, 3.0 and 5.0 wt.%).

**Figure 4:** SEM images of pure P(VDF-HFP) and P(VDF-HFP)/PANI composite nanofibers with different PANI concentrations at (**top**) 1000× and (**bottom**) 10,000× magnifications.

**Figure 5:** (**a**) XRD patterns and (**b**) FTIR spectra of pure P(VDF-HFP) and P(VDF-HFP)/PANI composite nanofibers with different PANI concentrations (0, 0.5, 1.0,1.5, 3.0 and 5.0 wt.%).

The article "Electrostrictive and Structural Properties of Poly(Vinylidene Fluoride-Hexafluoropropylene) Composite Nanofibers Filled with Polyaniline (Emeraldine Base)" was published in 2021. Journal: Polymers (Basel).

**Figure 6:** DMA curves of pure P(VDF-HFP) and P(VDF-HFP)/PANI composite nanofiber as a function of temperature; observed (**a**) storage modulus, (**b**) loss modulus, (**c**) tan delta, (**d**) stress–strain curves and (**e**) Young’s modulus of the samples versus weight fraction of PANI.

**Figure 7:** (**a**) Dielectric constant; (**b**) strain as a function of electric field at 1 Hz and (**c**) strain as a function of E^2^ for pure and P(VDF-HFP)/PANI composite nanofibers.

**Table 1:** Evaluated average diameter, water contact angle and elements of the samples.

P(VDF-HFP)/PANI Concentrations	Average Diameter (nm)	Water Contact Angle (Degree)	Element	
			F (%)	C (%)
0.00%	120.3 ± 20.6	139.2 ± 3.2°	55.5	44.5
0.50%	265.5 ± 53.1	132.6 ± 4.7°	53.3	46.7
1.00%	286.3 ± 72.7	131.9 ± 5.3°	54.5	45.5
1.50%	292.1 ± 50.2	130.4 ± 4.4°	55.9	44.1
3.00%	293.6 ± 32.9	130.2 ± 3.2°	55.0	45.0
5.00%	326.5 ± 99.5	126.8 ± 2.8°	51.8	48.2

**Table 2:** Evaluated crystallinity and β-phase fraction in the samples.

P(VDF-HFP)/PANI Concentrations	*X_c_* (%)	*A_β_*	*A_α_*	*F*(*β*) (%)	*%β* (%)
0.0%	48.40	0.2120	0.0605	73.53	35.59
0.5%	52.63	0.2477	0.0325	85.79	45.15
1.0%	55.58	0.2542	0.0300	87.03	48.37
1.5%	53.09	0.2583	0.0237	89.64	47.59
3.0%	55.91	0.2113	0.0217	88.53	49.50
5.0%	55.49	0.2123	0.0203	89.22	49.51
PANI	46.88	0.0582	0.0281	62.12	29.12

**Table 3:** Evaluated dielectric constant ($\varepsilon_{r}$), loss tangent, conductivity (*σ*), Young’ modulus (*Y*) and electrostrictive coefficient (*M_33_*) of pure and P(VDF-HFP)/PANI composites.

P(VDF-HFP)/PANI Concentrations	$\varepsilon_{r}$ at 100 Hz	*Loss Tangent* at 100 Hz	*σ* at 100 Hz (×10^−10^ S/m)	*Y* (MPa)	*M*_33_ (×10^−14^ m^2^/V^2^)	$\frac{\varepsilon_{r}\varepsilon_{0}}{Y}$
0.0%	1.48	0.00071	1.28	5.0 ± 1	1.28	2.62 × 10^−18^
0.5%	1.56	0.00086	2.98	22.5 ± 3	1.30	6.14 × 10^−19^
1.0%	1.92	0.00175	3.34	35.0 ± 2	1.73	4.86 × 10^−19^
1.5%	2.23	0.01542	4.34	40.0 ± 2	2.21	4.94 × 10^−19^
3.0%	2.28	0.01962	6.01	45.0 ± 3	2.42	4.49 × 10^−19^
5.0%	2.58	0.02403	9.18	50.0 ± 3	2.53	4.57 × 10^−19^

## Data Availability

Data availability upon request.
